RETRACTED

# Alisol B 23-Acetate Increases the Antitumor Effect of Bufalin on Liver Cancer through Inactivating Wnt/*β*-Catenin Axis

**DOI:** 10.1155/2022/6249534

**Published:** 2022-05-06

**Authors:** Miaoqing Ye, Yinghui Tang, Jinyu He, Xueyan Cao, Jiaojiao Liu, Shaojie Kou, Yueqing Yang, Jingdong Xue, Fenping Li

**Affiliations:** Department of Liver Disease, Shaanxi Provincial Hospital of Chinese Medicine, Xi'an, 710003 Shaanxi Province, China

## Abstract

**Objective:**

Liver cancer seriously threatens the health of people. Meanwhile, it has been reported that bufalin could act as an inhibitor in liver cancer. In addition, alisol B 23-acetate is a natural product derived from *Alisma plantago-aquatica Linn* which has an antitumor effect. In this study, we aimed to explore whether alisol B 23-acetate could increase the antitumor effect of bufalin on liver cancer.

**Methods:**

In order to detect the effect of alisol B 23-acetate in combination with bufalin on liver cancer, human liver cancer SMMC-7721 and MHCC97 cells were used as subjects. Bufalin and alisol B 23-acetate were performed on cells. Cell viability was tested by MTT assay. In addition, flow cytometry was performed to assess the cell apoptosis. Autophagy-related protein levels were tested by western blotting.

**Results:**

The data revealed that bufalin significantly decreased the viability of liver cancer cells, and the inhibitory effect was further increased by alisol B 23-acetate. In addition, alisol B 23-acetate notably enhanced the apoptotic effect of bufalin on liver cancer cells through mediation of Mcl-1, Bax, Bcl-2, and cleaved caspase-3. Meanwhile, alisol B 23-acetate in combination with bufalin induced the autophagy in liver cancer cells through mediation of Beclin-1 and p62. Furthermore, alisol B 23-acetate in combination with bufalin significantly downregulated the level of GSK-3*β* and increased the expression of *β*-catenin in liver cancer cells.

**Conclusion:**

In summary, these findings provide the first evidence that alisol B 23-acetate improves the anticancer activity of bufalin on liver cancer through activation of the Wnt/*β*-catenin axis, and these outcomes might shed new lights on exploring the new methods against liver cancer.

## 1. Introduction

Liver cancer (LC) is a frequent malignancy which has high incidence and mortality according to the previous report [1]. In addition, hepatocellular carcinoma (HCC) stands up for over 85% of primary LC, and it often results from the progression of chronic liver disease with the stimulation from environmental factors [2]. The outcomes of LC remain unsatisfactory irrespective of constant efforts made to the research of LC. Hence, it is pressing to explore new treatments of LC. Bufalin, isolated from traditional Chinese medicine, is the main digoxin-like immunoreactive component of Chansu [3]. Bufalin and other bufalene lactones are C-24 steroids with cardiac activity. They have a variety of biological activities, such as cardiac rigidity, anesthesia, blood pressure stimulation, respiration, and antitumor activities. Bufalin has been confirmed to exert antitumor action on multiple cancers. For instance, Zou et al. found the ability of bufalin to inhibit gastric cancer progression via modulating MAPK axis and Jin et al. revealed that bufalin could reduce NSCLC cell migration through modulation of the circ_0046264/miR-522-3p axis [4, 5]. Meanwhile, it has been reported that bufalin had inhibitory effects on LC; but, it would be great if the therapeutic efficacy of bufalin on LC could be further enhanced [6].

RETRACTED

Alisol B 23-acetate (AB23A) is a tetracyclic triterpenoid isolated from the rhizomes of Alisma orientalis which is a medicinal plant formulated into different traditional Chinese herbal medicine formulas [7]. In recent years, it has been revealed to biologically characterize and has several pharmacological activities, such as antihepatitis virus [8], antibacterial [9], and liver protection [10]. Liu et al. [11], for example, indicated that AB23A induced NSCLC cell apoptosis via the PI3K/Akt pathway inactivation; Zhao et al. suggested that AB23A induced colon cancer cell apoptosis through inducing autophagy induction [12]. Furthermore, AB23A could attenuate LC progression [13, 14]. However, whether it is capable of increasing the antitumor action of bufalin remains largely unknown.

The significant regulatory role of the Wnt/*β*-catenin axis in tumor progression has been well documented [15, 16]. The Wnt/*β*-catenin axis activation is reported to increase PTEN levels in bladder cancer *in vivo*, which leads to tumorigenesis when PTEN is genetically lost [17]. Furthermore, the Wnt/*β*-catenin axis has been demonstrated to have a close connection with the biological processes involved in cancer [18, 19]. Recently, AB23A has been reported to induce human osteosarcoma cell apoptosis through Wnt/*β*-catenin signal activation [20]. However, the research regarding the involvement of bufalin or AB23A in LC via the Wnt/*β*-catenin axis remains scarce. Based on the above backgrounds, the novelty and motivation of the study is to investigate whether AB23A in combination with bufalin can be an efficient treatment approach for LC and is the effect mechanism through Wnt/*β*-catenin signal activation. This study probes into the impact of AB23A in combination with bufalin on LC, in the hope of shedding new lights on exploring new treatments for LC.

RETRACTED

## 2. Materials and Methods

### 2.1. Cell Lines and Cell Culture

Supplied and authenticated by the Chinese Academy of Sciences, Shanghai, human LC cell strains SMMC-7721 and MHCC97 were cultivated in the 1640 complete medium (Gibco® Thermo Fisher Scientific Inc., Rockford, IL, USA) comprising 1% penicillin-streptomycin solution (Hyclone™, GE Healthcare Life Sciences, Utah, USA)+10% fetal bovine serum. The incubation was performed in a 5% CO_2_ incubator at 37°C in a humidified atmosphere.

### 2.2. Drug Treatment

After solubilization, bufalin (Selleck Co. LLC., St. Louis, USA) was stored at a concentration of 10 mM in 13% ethanol at 4°C, followed by dilution in the medium for use. The final concentration of ethanol was made <0.01%, so as not to influence cell growth or viability. Similarly, AB23A (Shanghai Yuanye Pharmaceutical Co., Ltd., Shanghai, China) was subjected to solubilization, storage at a concentration of 25 mM in sterile water at -20°C, and subsequent dilution in the medium before use. SMMC-7721 and MHCC97 cells were treated with serial dilutions of bufalin and/or AB23A and incubated for 24 and 48 h.

### 2.3. Cell Viability Analysis

Cell viability measurement was performed using the colorimetric MTT (Sigma) method, which quantified the reduction of yellow tetrazolium salt to purple formazan crystals by the mitochondria of live cells [21]. Cells adjusted to 5000 cells/per well were planted overnight in the wells of 96-well plates. Subsequently, they were intervened by AB23A (25, 50, 100, and 200 *μ*M) [12] and/or bufalin (25, 50, 100, and 200 *μ*M) [22] for 24, 48, or 72 h, followed by the addition of MTT solution to each well for 2 h. Afterwards, the cell supernatants were removed but added with DMSO into each well. Absordance (490 nm) was measured by a microplate reader (Thermo, Multiskan GO, USA).

### 2.4. Annexin-V Assay

After trypsinization, LC cells were treated with rinsing by phosphate-buffered saline and resuspension in Annexin V Binding Buffer. Then, they were subjected to 15 min of staining with 5 *μ*L FITC and 5 *μ*L propidium (PI) in the darkness. Annexin V-FITC/PI kit was purchased from Procell (Wuhan, China). The cell apoptosis rate was determined with the use of a flow cytometer (BD, Franklin Lake, NJ, USA).

### 2.5. 41,6-Diamidino-2-Phenylindole (DAPI) Staining

To assess the extent of apoptosis, nuclear morphology of SMMC-7721 and MHCC97 cells was evaluated using DAPI staining and observed using fluorescence microscopy (Olympus, Japan). Both cell lines (3 × 10^5^ cells/well) were planted onto 6-well plates and cultivated for 24 h with AB23A and/or bufalin. After treatment, they were treated with PBS washing and 30 min of paraformaldehyde (4%) fixation, followed by another PBS rinsing and nucleus staining with DAPI (2.5 *μ*g/mL). Fluorescence signals were photographed using an inverted Olympus IX71 microscope (Japan).

RETRACTED

### 2.6. Western Blotting Analysis

RIPA-extracted total protein from cell lysates or tissues was subjected to concentration determination with a BCA protein kit (Thermo Fisher Scientific). Proteins (40 *μ*g/lane) were then treated with 10% SDS-PAGE isolation and subsequent transfer onto polyvinylidene fluoride (Thermo Fisher Scientific) membranes. After a 1-hour blocking with 5% nonfat-dried milk, the membranes were immersed in *Ι* antibodies for overnight cultivation (4°C). Thereafter, they were immersed in a II anti-rabbit antibody (HRP-conjugated, ab7090; 1 : 5000) for another 1 h of cultivation at ambient temperature. Membrane scanning was performed via an Odyssey Imaging System and analyzed using Odyssey *v*2.0 (LICOR Biosciences, Lincoln, NE, USA). The *Ι* antibodies included the following (all diluted at 1 : 1000 and supplied by Cell Signaling Technologies, Beverly, MA): anti-Mcl-1 (#94296), anti-Bcl-2 (#15071), anti-caspase-3 (#9662), anti-Bax (#14796), anti-Beclin-1 (#4122), anti-p62 (#8025), anti-LC3 (#3868), anti-GSK-3*β* (#12456), anti-*β*-catenin (#8480), and anti-*β*-actin (#3700). *β*-Actin was considered an internal control.

### 2.7. Statistical Analysis

All experimental data were the average of at least 3 independent tests. Analysis of experimental data (mean ± SD) was done by GraphPad Prism *v*6.00 for Windows (GraphPad Software, La Jolla California USA, http://www.graphpad.com). One-way or two-way ANOVA was responsible for all the statistical analyses in this research, followed by Dunnett's multiple comparisons test, with the difference considered significant at a *p* value of 0.05.

## 3. Results

### 3.1. AB23A Increases the Antiproliferative Effect of Bufalin on LC Cells

To test the impacts of AB23A or/and bufalin on LC cell viability, SMMC-7721 and MHCC97 cell viabilities were determined by MTT assay after treatment with AB23A or bufalin of the above indicated concentrations. As shown in Figures 1(a)–1(d), AB23A or bufalin decreased LC cell viability in a dose- and time-dependent fashion. In addition, bufalin's influence on LC cell viability was further increased by AB23A (Figures 1(e) and 1(f). The data suggest enhanced antiproliferative effects of bufalin by AB23A on LC cells.

### 3.2. AB23A and/or Bufalin Induced LC Cell Apoptosis

Flow cytometry was utilized for the assessment of the impacts of AB23A/bufalin on LC cell apoptosis. As indicated in Figures 2(a) and 2(b), AB23A or bufalin significantly induced LC cell apoptosis, and bufalin-induced cell apoptosis was further increased after the addition of AB23A. Besides, Bax and cleaved caspase-3 were notably elevated in LC cells by AB23A or bufalin, and the combination treatment (AB23A plus Bufalin) exhibited the better effect (Figures 3(a) and 3(b)). In contrast, AB23A or bufalin notably downregulated the levels of Mcl-1 and Bcl-2, and more marked downregulation was observed when AB23A and bufalin were used together (Figures 3(a) and 3(b)). In summary, AB23A and/or bufalin induced the apoptosis in LC cells through mediation of Bax, Bcl-2, cleaved caspase-3, and Mcl-1.

RETRACTED

### 3.3. Combination of AB23A and Bufalin Induces LC Cell Autophagy

To investigate the effect of AB23A/bufalin on LC cell autophagy, we investigated autophagy-related proteins (Beclin-1, p62, and LC3 II/I) using western blotting. The data revealed that AB23A or bufalin significantly upregulated Beclin-1 and LC3 II/I and declined p62 in LC cells (Figures 4(a) and 4(b)). Furthermore, the combination treatment further increased the influence of AB23A or bufalin alone (Figures 4(a) and 4(b)). All these results suggest enhanced autophagy-inducing effects of bufalin by AB23A in LC cells.

### 3.4. AB23A and/or Bufalin Inhibited LC Progression via Wnt/*β*-Catenin Axis Inactivation

We intervened LC cells with bufalin and/or AB23A to explore whether the Wnt/*β*-catenin axis plays a similar role in AB23A/bufalin-induced apoptosis in LC. As presented in Figures 5(a) and 5(b), AB23A or bufalin significantly downregulated GSK-3*β* but increased *β*-catenin in LC cells (Figures 5(a) and 5(b)). In order to verify whether the inhibition of Wnt/*β*-catenin by AB23A/bufalin combination affected LC cell viability, we treated both cell lines with different concentrations of XAV939, a Wnt/*β*-catenin inhibitor. XAV939 was found to dose dependently decrease LC cell viability (Figures 5(a) and 5(b)). This indicated that AB23A/bufalin combination hinders LC cell viability by inducing cell death through activating Wnt/*β*-catenin signaling (Figures 5(c) and 5(d)). To sum up, AB23A and/or bufalin inhibited LC progression via Wnt/*β*-catenin axis inactivation.

## 4. Discussion

Bufalin is a commonly used drug for patients with LC. However, although effective, bufalin has been known for causing side effects and risks. After a short period of response, most patients develop therapeutic resistance and tumors usually relapse. Therefore, the development of new treatment options is urgently needed to overcome side effects and drug resistance and to improve efficacy. Based on our increased understanding of the molecular mechanisms of tumor growth, rational combination regimens may be conducive to improving the median survival of LC patients. In this research work, we investigated the efficacy of AB23A in combination with bufalin on LC cells.

RETRACTED

The ability of AB23A to inhibit LC cell growth was in agreement with previous reports [23–25]. In addition, we identified that AB23A inhibits the growth of SMMC-7721 and MHCC97, both of which are LC cell strains. Previous studies indicated that these two cell lines are used to represent the drug-resistant LC cells [26, 27]. The research is aimed at investigating how and whether AB23A can improve the anticancer activity of bufalin against LC cells. We further demonstrated that AB23A and bufalin could inhibit SMMC-7721 and MHCC97 cell growth in a dose- and time-dependent fashion, and this was in conformity with previous literature. Our data suggested that dose and schedule optimization of AB23A may be conducive to enhancing the antitumor activity of bufalin and that in future bufalin combination clinical trials, a combination therapy with a rational dosage of AB23A may contribute to better efficacy compared with increasing the dose of bufalin on a monotherapy basis. The combination with AB23A reduced SMMC-7721 and MHCC97 cell viability and increased bufalin sensitivity and cellular cytotoxicity. The results showed that AB23A enhanced the efficacy of bufalin, which is one of the agents that target microtubules, in the SMMC-7721 and MHCC97 cells *in vitro*. Apoptosis results primarily from the ‘extrinsic' or ‘intrinsic' caspase-dependent pathways of cell death, including mitogen-activated protein kinase, mTOR pathway, or PI3K/Akt pathways [28]. Reportedly, the pro- and antiapoptotic Bcl-2 family members may play a role in this interaction. In LC cells, three common antiapoptotic Bcl proteins Bcl-xl, Bcl-2, and Mcl-1, as well as proapoptotic protein Bax, were identified. Bcl-2 family inhibition can sensitize SMMC-7721 cells to bufalin, revealing a unique apoptosis pathway in which members of the Bcl-2 family trigger caspase-dependent cell apoptosis in LC cells [29, 30]. Mcl-1 overexpression has a connection with advanced LC, including advanced Gleason grade primary and metastatic tumors. Thus, Mcl-1, which is modulated at multiple levels, has been identified as an essential regulatory factor of cell survival [31]. Moreover, the metformin/aspirin combination was found to significantly inhibit pancreatic cancer cell proliferation by decreasing the expression of Mcl-1 and Bcl-2 [32]. The multilevel modulation highlights the role of Mcl-1 as a critical regulator of apoptosis and a potential biomarker. Previous studies showed that AB23A induces apoptosis of androgen-independent human prostate cancer cells via the mitochondrial pathway and caspase (caspase-3, caspase-8, and caspase-9) activation [33, 34]. Caspase activation is an important pathway for apoptosis signaling, which directly induces eventual apoptosis events [35]. Here, our results indicated that AB23A+bufalin significantly promoted cell apoptosis compared with their single use in SMMC-7721 and MHCC97 cells. It is stated that AB23A promotes bufalin-induced apoptosis but AB23A alone readily induces much more apoptosis than bufalin. Therefore, AB23A may have higher sensitization effect on SMMC-7721 and MHCC97 cells than bufalin. Furthermore, we also reported that AB23A+bufalin distinctly decreased Mcl-1 and upregulated cleaved caspase-3 and Bax/Bcl-2 ratio compared to either AB23A or bufalin alone, indicating that promoted downregulation of Mcl-1 might have enhanced caspase-3 and Bax/Bcl-2-dependent apoptosis and potentially playing a role in this interaction. Also, when analyzing apoptosis, we observed that Bax/Bcl-2 ratios in SMMC-7721 and MHCC97 cells.

RETRACTED

Drug resistance is a complex process composed of many factors such as abnormal apoptosis and autophagy, which affect cancer chemosensitivity [36]. Autophagy, or type II programmed cell death, interferes with the onset and progression of a wide spectrum of diseases and has intricate interactions with apoptosis [37]. Autophagy can inhibit the occurrence of HCC, but autophagy occurs when liver cancer cells are damaged by hypoxia, drugs, or toxic chemicals [38]. Studies have shown that the important regulatory role of Beclin-1 gene in autophagy is mainly through the interaction of its own BH3 domain with Bcl-2 family proteins [39]. It has been reported that apart from antiapoptotic effects, Bcl-2 also binds to Beclin-1 to inhibit autophagy activation [40]. Furthermore, Mcl-1 degradation was also found to be an initiating event for autophagy activation. Germain et al. found that AB23A upregulated Beclin-1 expression and LC3 II/I level to induce autophagy in human osteosarcoma cells [41]. Here, the similar results were obtained in this study. Our findings suggested that AB23A+bufalin significantly increased Beclin-1 expression and LC3 II/I ratio compared with their single use, indicating that both can promote autophagy of SMMC-7721 and MHCC97 cells. Meanwhile, Sheng et al. [42] have found that bufalin induced cell autophagy and inhibited proliferation of liver cancer cells by influencing the expression of autophagy-related proteins in liver cancer cells and the autophagic state of liver cancer cells affected the inhibitory effect of bufalin on the proliferation of liver cancer cells.

RETRACTED

The precise molecular mechanism by which AB23A potentiates bufalin remains to be elucidated. Abnormal activation of the Wnt/*β*-catenin axis has a close connection with the development of many human tumors like prostate cancer [43, 44]. Ma et al. reported that AB23A induced human osteosarcoma cell apoptosis through Wnt/*β*-catenin signal activation [20]. However, the impacts of AB23A+bufalin on the Wnt/*β*-catenin axis in LC cells have not been studied so far. Normally, the cytosolic *β*-catenin protein forms a “degradation complex” with Axin, APC, GSK-3, and CK1 and is phosphorylated to form a phosphorylated *β*-catenin protein, which is recognized and degraded by the ubiquitin-linked enzyme *β*-TrCP, thereby failing to activate its target gene [45, 46]. This study showed that AB23A in combination with bufalin increased *β*-catenin protein, while decreased GSK-3*β* in LC cell strains (SMMC-7721 and MHCC97), suggesting the ability of AB23A and bufalin to activate the Wnt/*β*-catenin axis. The results were similar to the previous studies that AB23A activates the Wnt/*β*-catenin axis in human osteosarcoma cells by downregulating GSK-3*β* and upregulating *β*-catenin [20].

## 5. Conclusion

Our study presents some limitations. First, since caspase-dependent apoptosis is involved, the mitochondrial dysfunction should be confirmed using appropriate experiments such as reduction of mitochondrial *trans*-membrane potential (delta psim). In addition, animal studies are needed for investigating the potential of AB23A/bufalin *in vivo*. The connection between drug(s)-induced apoptosis or autophagy and Wnt/*β*-catenin signal activation remains to be investigated. Thus, the planning of our future research is to validate the mutual regulation of apoptosis and autophagy and its association with the Wnt/*β*-catenin axis. The impacts of AB23A and bufalin on LC cell stains SMMC-7721 and MHCC97 were discussed in the present work. Our data indicate that AB23A significantly potentiates bufalin in treating LC via Wnt/*β*-catenin signal inactivation, which provides novel ideas for LC treatment. Although our results were performed *in vitro*, the prospect of our study is to further conduct it to confirm the effectiveness and safety of AB23A in combination with bufalin in vivo and apply it to the clinical trials to provide a treatment approach in liver cancer.

## Figures and Tables

**Figure 1:** Alisol B 23-acetate increases the antiproliferative effect of bufalin on liver cancer cells. (a) Effect of bufalin treatment on the viability of SMMC-7721 cells. (b) Effect of bufalin treatment on the viability of MHCC97 cells. (c) Effect of alisol B 23-acetate alone on the viability of SMMC-7721 cells. (d) Effect of alisol B 23-acetate alone on the viability of MHCC97 cells. (e) Effect of alisol B 23-acetate in combination with bufalin on the viability of SMMC-7721 cells. (f) Effect of alisol B 23-acetate in combination with bufalin on the viability of MHCC97 cells. Error bars represent the SD (*n* = 5). Compared with the control group, ^∗∗^*p* < 0.01; compared with the bufalin or alisol B 23-acetate group, ^##^*p* < 0.01.

RETRACTED

**Figure 2:** Alisol B 23-acetate and/or bufalin induced the apoptosis in liver cancer cells. (a) Representative flow cytometry with Annexin V/PI plots in SMMC-7721 cells. (b) Representative flow cytometry with Annexin V/PI plots in MHCC97 cells. Summary of apoptosis rate obtained from flow cytometry was presented for each cell line. Apoptosis was evaluated as the sum of primary apoptosis (Q3 quadrant) and late apoptosis (Q2 quadrant). Error bars represent the SD (*n* = 3). Compared with the control group, ^∗∗^*p* < 0.01; compared with the bufalin or alisol B 23-acetate group, ^##^p <0.01.

**Figure 3:** Alisol B 23-acetate in combination with bufalin induces the apoptosis in liver cancer cells via mediation of Bax, cleaved caspase-3, Bcl-2, and Mcl-1. (a) The expression levels of Mcl-1, Bax, Bcl-2, and cleaved caspase-3 in SMMC-7721 cells were measured by western blotting. (b) Expression of Mcl-1, Bax, Bcl-2, and cleaved caspase-3 in MHCC97 cells were measured by western blotting. Error bars represent the SD (*n* = 5). Compared with the control group, ^∗∗^*p* < 0.01; compared with the bufalin or alisol B 23-acetate group, ^##^*p* < 0.01.

**Figure 4:** Combination of alisol B 23-acetate and bufalin induces the autophagy in liver cancer cells. (a) The expression levels of Beclin-1, p62, and LC3 II/I in SMMC-7721 cells were measured by western blotting. (b) Expression of Beclin-1, p62, and LC3 II/I in MHCC97 cells were measured by western blotting. Error bars represent the SD (*n* = 5). Compared with the control group, ^∗∗^*p* < 0.01; compared with the bufalin or alisol B 23-acetate group, ^##^*p* < 0.01.

**Figure 5:** Alisol B 23-acetate and/or bufalin inhibited the progression of liver cancer via inactivation of the Wnt/*β*-catenin axis. (a) The expression levels of GSK-3*β* and *β*-catenin in SMMC-7721 cells. (b) The expression levels of GSK-3*β* and *β*-catenin in MHCC97 cells. (c) The effect of the Wnt/*β*-catenin signaling inhibitor XAV939 (20 *μ*M) on the cell viability of SMMC-7721 cells. (d) The effect of the Wnt/*β*-catenin signaling inhibitor XAV939 (20 *μ*M) on the cell viability of MHCC97 cells. Error bars represent the SD (*n* = 5). Compared with the control group, ^∗∗^*p* < 0.01; compared with the bufalin or alisol B 23-acetate group, ^##^*p* < 0.01.

RETRACTED

## Data Availability

All data generated or analyzed during this study are included in this published article.
